The article "Adaptive Fuzzy Sliding Mode Control of a Pressure-Controlled Artificial Ventilator" was published in 2021. Journal: J Healthc Eng.

# Adaptive Fuzzy Sliding Mode Control of a Pressure-Controlled Artificial Ventilator

**DOI:** 10.1155/2021/1926711

**Published:** 2021-06-23

**Authors:** Ibrahim M. Mehedi, Heidir S. M. Shah, Ubaid M. Al-Saggaf, Rachid Mansouri, Maamar Bettayeb

**Affiliations:** ^1^Department of Electrical and Computer Engineering (ECE), King Abdulaziz University, Jeddah 21589, Saudi Arabia; ^2^Center of Excellence in Intelligent Engineering Systems (CEIES), King Abdulaziz University, Jeddah 21589, Saudi Arabia; ^3^Laboratoire de Conception et Conduite des Systemes de Production (L2CSP), Tizi-Ouzou 15000, Algeria; ^4^Electrical Engineering Department, University of Sharjah, Sharjah, UAE

## Abstract

This paper presents the application of adaptive fuzzy sliding mode control (AFSMC) for the respiratory system to assist the patients facing difficulty in breathing. The ventilator system consists of a blower-hose-patient system and patient's lung model with nonlinear lung compliance. The AFSMC is based on two components: singleton control action and a discontinuous term. The singleton control action is based on fuzzy logic with adjustable tuning parameters to approximate the perfect feedback linearization control. The switching control law based on the sliding mode principle aims to minimize the estimation error between approximated single fuzzy control action and perfect feedback linearization control. The proposed control strategy manipulated the airway flow delivered by the ventilator such that the peak pressure will remain under critical values in presence of unknown patient-hose-leak parameters and patient breathing effort. The closed-loop stability of AFSMC will be proven in the sense of Lyapunov. For comparative analysis, classical PID and sliding mode controllers are also designed and implemented for mechanical ventilation problems. For performance analysis, numerical simulations were performed on a mechanical ventilator simulator. Simulation results reveal that the proposed controller demonstrates better tracking of targeted airway pressure compared with its counterparts in terms of faster convergence, less overshoot, and small tracking error. Hence, the proposed controller provides useful insight for its application to real-world scenarios.

## 1. Introduction

Several new viruses, epidemics, and even pandemics have emerged in the past 20 years. 774 people have been killed by the severe acute respiratory syndrome (SARS) that first emerged in mid-November 2002 in the Guangdong province, China [1]. In 2009, the World Health Organization (WHO) had declared a new global pandemic called H1N1 influenza. Although the confirmed number of deaths by WHO are 18,500, Dawood [2] in his studies estimates the actual number should be between 151,700 and 575,400. The most recent is the Middle East respiratory syndrome (MERS-CoV) in 2012 with 806 associated deaths reported in December 2018 mostly in Saudi Arabia [3]. Before the pandemic COVID-19 where to date, over 50 million people have been contacted with the disease with over 1 million deaths recorded since its discovery in the Wuhan province, China, in December 2019. The common cause of death for patients who contracted these diseases are acute respiratory distress syndrome (ARDS) where according to a study, 40 percent of critically ill COVID-19 patients developed this respiratory failure [4–7]. In most cases of ARDS, patients will have to be supported with mechanical ventilation to assist or replace their spontaneous breathing [8].

The article "Adaptive Fuzzy Sliding Mode Control of a Pressure-Controlled Artificial Ventilator" was published in 2021. Journal: J Healthc Eng.

The earliest usage of mechanical ventilators as a device to provide ventilatory assistance can be traced back to the 18th century. However, it was only in the 1950s that the first closed-loop system for mechanical ventilation was introduced. During this time, mechanical bellows and valves were used in mechanical ventilators to cycle gas into the lung, while pneumatic components were used to implement simple proportional (P) or proportional integral (PI) controller [9]. Microprocessors were eventually used to implement those controllers, and since then, many types of closed-loop controls have been proposed.

Walter and Leonhardt [10] classify the different levels of automatic control in artificial ventilation into three categories according to the amount of interaction between the patient and medical devices. In class 1 control loops called *device-internal control loops* and class 2 control loops called *patient-oriented control loops*, control signals are measured inside the device. The difference between both classes is that the interaction between the patient and device is possible in class 2, while there are no such features in class 1 control loops. Instead of using physical parameters, a class 3 control loop used physiological parameters as its control variable and for that it is called *physiological compensatory control loops*. In this paper, a pressure-based ventilation controller under the class 2 category is developed where the control objective is to track a set-point of target airway pressure.

One type of controller that has been used widely in mechanical ventilation is the PID controller. One of its earliest implementation since the introduction of the microprocessor can be found here [11]. This type of controller is however known for its poor performance on a system where its dynamic is not constant, which is the case for mechanical ventilation. The lung compliance and resistance are two parameters in the mechanical ventilation system that are changing according to the lung volumes and are different from patient to patient. Many researchers have proposed improvement to the PID controller in mechanical ventilation, which includes the addition of an adaptive mechanism [12], an optimization technique [13], and automatic tuning of PID gains [14].

The article "Adaptive Fuzzy Sliding Mode Control of a Pressure-Controlled Artificial Ventilator" was published in 2021. Journal: J Healthc Eng.

The accurate information of the system dynamics is quite essential for designing nonlinear control systems. Model-based controllers [15, 16] are employed, which are more transparent as they are developed from the mathematical models derived from physiological processes. A slight disadvantage could be in obtaining the precise mathematical model required for a good performance especially as patient dynamics are uncertain, which is the same case as inverse dynamic controller [17]. Other types of controller implemented in mechanical ventilation from our literature searches are model predictive control [18], variable-gain control [19], and repetitive control [20].

There are nonlinear control strategies available in the literature that does not require exact knowledge of the system dynamics [21, 22]. Among these controllers, sliding mode control (SMC) is a powerful method with inherited robust attitudes to control complex dynamical systems [23, 24]. However, conventional SMC may potentially experience chattering problems in the control command, which degrades the control performance by exciting unmodeled high-frequency dynamics, which may lead to instability [25]. Noninteger control, or fractional-order control (FOC), has received significant attention in control engineering due to its ability to tune time-varying systems while remaining controllable [26, 27]. Noninteger calculus significantly improves the performance of PID controllers. The fact has been investigated in previous studies [26–29].

In literature, fuzzy logic control (FLC), which falls under the category of intelligent control, has been widely used as an alternative to control the nonlinear system in presence of unknown dynamics and external perturbations [30, 31]. There were also attempts of using FLC in mechanical ventilation [32, 33], which is easy to implement as it does not require explicit mathematical models. However, traditional FLC may require some systematic mechanism for mapping the expert knowledge into the rule base of fuzzy interference system [34, 35]. Hence, the subject control strategy could have limited transparency. Thus, extensive testing with hardware will be required for its validation and verification such that closed-loop stability is guaranteed. To cope with this, it is preferable to augment some adaptive mechanism for adjusting the control parameters automatically while guaranteeing closed-loop stability. In adaptive fuzzy, there are two widely used control approaches: direct and indirect. The former approach is based on adjusting the control parameters with changing dynamics, whereas the later indirect approach is responsible to identify the unknown system parameters [4]. As a result, both of these strategies are striving to achieve the desired system performance by adjusting the fuzzy rules accordingly [36–39].

The article "Adaptive Fuzzy Sliding Mode Control of a Pressure-Controlled Artificial Ventilator" was published in 2021. Journal: J Healthc Eng.

In literature, various combinations of SMC and FLC have been proposed to handle complex and unmodeled dynamics [40, 41] and have been applied to various nonlinear systems [42–44] including microelectromechanical system (MEMS) resonators [45]. In prior studies [46–48], the authors have implemented fuzzy double hidden layer recurrent neural network to approximate the SMC-based equivalent control, eliminating the unknown disturbance while reducing the impact of switching gain. Similarly, Poursamad and Davaie-Markazi [49] have implemented a variant of hybrid FLC and SMC control titled robust adaptive fuzzy control for Duffing oscillators and atomic force microscopes. The later methodology has been adopted in this article to approximate the ideal control law based on fuzzy approximation theory while handling modeling uncertainties and disturbances through augmentation of SMC-based switching control law.

This paper deals with a design of direct form of adaptive fuzzy sliding mode control (AFSMC) by exploiting the potential of both SMC and FLC strategies to handle complex and unmodeled dynamics. The resultant control expression comprised singleton fuzzy control action, which adjusts itself based on Lyapunov energy function, and switching control element, which aims to minimize the approximation error between fuzzy control and perfect feedback linearization control law. The resultant controller drastically enhances the robustness while guaranteeing the asymptotic stability of the closed-loop system. As a case study, the proposed AFSMC controller is employed for pressure control of the well-known mechanical ventilator system. To visualize the performance attributes, a simulation model of the mechanical ventilator system is modeled in Simulink/MATLAB environment. Numerical simulations reveal that the direct form of AFSMC is quite effective by steering the pressure in the closed vicinity of the desired pressure curve.

The rest of this paper is organized as follows: the detailed mathematical modeling of ventilator system is given in Section 2. The description of AFSMC controller is presented in Section 3 with detailed stability proof in the sense of Lyapunov. Simulation results of AFSMC along with its comparison with classical PID and SMC are depicted in Section 4. Finally, the paper is concluded in Section 6.

The article "Adaptive Fuzzy Sliding Mode Control of a Pressure-Controlled Artificial Ventilator" was published in 2021. Journal: J Healthc Eng.

## 2. Artificial Ventilator Modeling

In this paper, a blower-hose-patient system model introduced in [50] consists of 3 main components—the blower, the hose, and the patient—is used to represent the respiratory system model as shown in Figure 1. The function of the blower is to generate the desired pressure *p*_*o*_ by compressing the atmospheric air, while the hose links the respiratory module to the patient. A single compartmental model presented in [19] is used to represent the patient's lung model. The aim of the controller is to track the airway pressure *p*_*aw*_ that is measured by a sensor positioned inside the module so that it follows the target set-point *p*_*t*_. With that, we can describe the error equation as follows:

(1) $$\begin{array}{c} e=p_{t}-p_{aw}. \end{array}$$

During the inhalation process, the patient will inhale the air from the blower (*Q*_*o*_) into the lung (*Q*_*p*_), then exhale back to the hose. To avoid the patient from taking the exhaled air back in the next cycle, a leak is positioned before the end of the tube to release the exhaled air (*Q*_leak_). Hence, we can write the patient flow dynamic as follows:

(2) $$\begin{array}{c} Q_{p}=Q_{o}-Q_{\text{leak}}. \end{array}$$

The airflow is derived from the pressure differences over resistance; thus, in this model, resistance in the hose (*R*_*h*_), in the leak (*R*_leak_), and in the patient's lung (*R*_*l*_) must also be taken into account. We can therefore describe the relationships between blower flow, leak flow, and patient flow with the resistances as follows:

(3) $$\begin{array}{c} Q_{o}=\frac{p_{o}-p_{aw}}{R_{h}}, \end{array}$$

(4) $$\begin{array}{c} Q_{\text{leak}}=\frac{p_{aw}}{R_{\text{leak}}}, \end{array}$$

(5) $$\begin{array}{c} Q_{p}=\frac{p_{aw}-p_{l}}{R_{l}}. \end{array}$$

The lung pressure can be depicted by the following differential equation:

(6) $$\begin{array}{c} {\dot{p}}_{l}=\frac{1}{C_{l}}Q_{p}, \end{array}$$

where *C*_*l*_ denotes the lung compliance. Combining equations (3)–(6) results in the following lung dynamics:

(7) $$\begin{array}{c} {\dot{p}}_{l}=\frac{p_{aw}-p_{l}}{C_{l}R_{l}}. \end{array}$$

We can derive the formula for airway pressure by substituting equations (3)–(5) into (2) as shown below:

(8) $$\begin{array}{c} p_{aw}=\frac{\left(1/R_{l}\right)p_{l}+\left(1/R_{h}p_{o}\right)}{\left(1/R_{l}\right)+\left(1/R_{h}\right)+\left(1/R_{\text{leak}}\right)}. \end{array}$$

The differential equation for the lung dynamic in (6) can now be rewritten by substituting the airway pressure expression in (8) into it as follows:

(9) $$\begin{array}{c} {\dot{p}}_{l}=\frac{-\left(\left(1/R_{h}\right)+\left(1/R_{l}\right)\right)p_{l}+\left(1/R_{h}\right)p_{o}}{R_{l}C_{l}\left(\left(1/R_{l}\right)+\left(1/R_{h}\right)+\left(1/R_{\text{leak}}\right)\right)}. \end{array}$$

We can represent (5), (7), and (8) in the state-space form as follows:

(10) $$\begin{array}{c} {\dot{p}}_{l}=A_{h}p_{l}+B_{h}p_{o}, \end{array}$$

(11) $$\begin{array}{c} \left[\begin{array}{c} p_{aw}\\ Q_{p} \end{array}\right]=C_{h}p_{l}+D_{h}p_{o}, \end{array}$$

where *p*_*o*_ is the input, [*p*_*aw*_, *Q*_*p*_]^*T*^ is the output vector, *p*_*l*_ is the state, and

(12) $$\begin{array}{c} A_{h}=-\frac{\left(1/R_{h}\right)+\left(1/R_{\text{leak}}\right)}{R_{l}C_{l}\left(\left(1/R_{l}\right)+\left(1/R_{h}\right)+\left(1/R_{\text{leak}}\right)\right)}, \end{array}$$

(13) $$\begin{array}{c} B_{h}=\frac{\left(1/R_{h}\right)}{R_{l}C_{l}\left(\left(1/R_{l}\right)+\left(1/R_{h}\right)+\left(1/R_{\text{leak}}\right)\right)}, \end{array}$$

(14) $$\begin{array}{c} C_{h}={\left[\frac{\left(1/R_{l}\right)}{\left(1/R_{l}\right)+\left(1/R_{h}\right)+\left(1/R_{\text{leak}}\right)}-\frac{\left(1/R_{h}\right)+\left(1/R_{l}\right)}{R_{l}\left(\left(1/R_{l}\right)+\left(1/R_{h}\right)+\left(1/R_{\text{leak}}\right)\right)}\right]}^{T}, \end{array}$$

(15) $$\begin{array}{c} D_{h}={\left[\frac{\left(1/R_{h}\right)}{\left(1/R_{l}\right)+\left(1/R_{h}\right)+\left(1/R_{\text{leak}}\right)}\frac{\left(1/R_{h}\right)}{R_{l}\left(\left(1/R_{l}\right)+\left(1/R_{h}\right)+\left(1/R_{\text{leak}}\right)\right)}\right]}^{T}. \end{array}$$

The blower system on the other hand can be represented by the following state-space model:

(16) $$\begin{array}{c} {\dot{x}}_{b}=A_{b}x_{b}+B_{b}P_{\text{con}}, \end{array}$$

(17) $$\begin{array}{c} p_{o}=C_{b}x_{b}. \end{array}$$

Finally, the complete general state-space model of the artificial ventilator is obtained by coupling expression in (10) with (16) and (17) as follows:

(18) $$\begin{array}{c} {\dot{x}}_{p}=\left[\begin{array}{c} {\dot{x}}_{b}\\ {\dot{p}}_{l} \end{array}\right]\\ =\left[\begin{array}{cc} A_{b} & 0\\ B_{h}C_{b} & A_{h} \end{array}\right]\left[\begin{array}{c} x_{b}\\ p_{l} \end{array}\right]+\left[\begin{array}{c} B_{b}\\ 0 \end{array}\right]P_{\text{con}}. \end{array}$$

The article "Adaptive Fuzzy Sliding Mode Control of a Pressure-Controlled Artificial Ventilator" was published in 2021. Journal: J Healthc Eng.

## 3. Design of AFSMC

This section presents the direct form of adaptive control employing FLC and SMC to achieve precise tracking performance while ensuring closed-loop stability of the mechanical ventilator. This has been accomplished by augmenting fuzzy approximation theory and principle of sliding mode control theory in the proposed AFSMC method, which proves to be robust against parametric uncertainties and perturbations.

### 3.1. Problem Statement

Consider the class of *n*th order control-affine nonlinear system given as

(19) $$\begin{array}{c} x_{n}=f\left(x,t\right)+g\left(x,t\right)u+d\left(t\right),\\ y=x, \end{array}$$

where *f*(**x**, *t*) and *g*(**x**, *t*) are the smooth and continuous bounded nonlinear functions, **x** ∈ *R*^*n*^ is the state vector assumed to be measurable, *u* ∈ *R* and *y* ∈ *R* are the control input and output of the system, respectively, and *d*(*t*) is the unknown but bounded disturbances such that *d*(*t*) ≤ *D*. If the state transition function *f*(**x**, *t*) and control input vector *g*(**x**, *t*) are perfectly known, then a perfect feedback linearization control law to follow the desired state trajectory *x*_*d*_ in presence of modeling uncertainties and exogenous disturbances is given by

(20) $$\begin{array}{c} u^{*}=\frac{1}{g\left(x,t\right)}\left[-f\left(x,t\right)+{\ddot{x}}_{d}-k_{1}\dot{e}\left(t\right)-k_{2}e\left(t\right)\right]. \end{array}$$

where *e*(*t*)=*x* − *x*_*d*_ is the tracking error, while *k*_1_ and *k*_2_ are the positive gain constants. However, in practice, it is not possible to determine the exact value of *f*(**x**, *t*) and *g*(**x**, *t*); therefore, it is difficult to apply control law given by (20). Hence, it is preferable to introduce some adaptive component in feedback linearization control law that will adjust the control parameters to improve tracking performance and to guarantee closed-loop stability.

### 3.2. AFSMC Design Based on Universal Approximation Theorem

This section presents the design of AFSMC control for pressure control of mechanical ventilator systems. The proposed control methodology integrates the fuzzy approximation theory and principles of sliding mode control into a fuzzy controller, which proves to be insensitive against modeling uncertainties and external perturbations. The decision-making capability of fuzzy control employing linguistic information has been proved to be effective for controlling nonlinear complex systems. The prime objective of the fuzzy controller is to approximate the pressure control command *P*_con_ such that it will approach the ideal control law *u*^*∗*^ given by (20) to arbitrary accuracy by defining multiple output fuzzy sets with singleton membership functions. With a view that the fuzzy rule base grows exponentially as the number of input variables increases, the sliding surface as a function of state variables is considered the input to the fuzzy set. The sliding surface being input to the fuzzy system is defined as

(21) $$\begin{array}{c} s\left(t\right)=\dot{e}\left(t\right)+k_{1}e\left(t\right)+k_{2}\int e\left(t\right)\text{d}t. \end{array}$$

where *e*(*t*)=*P*_*t*_ − *P*_*aw*_, *λ* is the Laplace operator, and the variables *k*_1_, *k*_2_, and *k*_3_ are the coefficients of Hurwitz polynominal *h*(*λ*)=*λ*^*n*−1^+*k*_*n*−1_*λ*^*n*−2^+⋯+*k*_1_, such that all the root lies in the open left half-plane. Taking the derivative of the sliding surface given by (21) implies

(22) $$\begin{array}{c} \dot{s}\left(t\right)=\ddot{e}\left(t\right)+k_{1}\dot{e}\left(t\right)+k_{2}e\left(t\right). \end{array}$$

To make the IF part of the input variable *s*, symmetric and uniformly distributed triangular membership functions are used, whereas the output of the fuzzy system *P*_*fz*_ is defined as the singleton control action *α*_*i*_, *i*=1,2,..,*n*, where *n* is the number of fuzzy rules as shown in Figure 2.

The article "Adaptive Fuzzy Sliding Mode Control of a Pressure-Controlled Artificial Ventilator" was published in 2021. Journal: J Healthc Eng.

The *i*th fuzzy linguistic rule involved the design process is written in the following form.

Rule *i*: If *s* is in the domain of *F*_*s*_^*i*^, then *P*_*fz*_*i*__ is *α*_*i*_.

The control law *P*_*fz*_ is obtained by the center of gravity defuzzification method [45], which implies

(23) $$\begin{array}{c} P_{fz}\left(\alpha ,\xi \right)=\frac{\sum_{i=1}^{m}\alpha_{i}\cdot \omega_{i}}{\sum_{i=1}^{m}\omega_{i}}, \end{array}$$

where *ω*_*i*_ is the firing strength of the *i*th rule. In order to cope with uncertain and complex unmodeled system dynamics, the singleton control action *α*_*i*_ is chosen to be an adjustable parameter with respect to changing environment [34]. The resultant adaptive fuzzy control law *P*_*fz*_ as a function of tunable parameter *α* can explicitly be expressed as

(24) $$\begin{array}{c} P_{fz}\left(\alpha ,\xi \right)=\alpha^{T}\xi , \end{array}$$

where the vector *α*=[*α*_1_, *α*_2_,…,*α*_*m*_]^*T*^ represents the parameter vector and *ξ*=[*ξ*_1_, *ξ*_2_,…,*ξ*_*m*_]^*T*^ symbolize the regressive vector, while *ξ*_*i*_ is defined as

(25) $$\begin{array}{c} \xi_{i}=\frac{\omega_{i}}{\sum_{i=1}^{m}\omega_{i}}. \end{array}$$

The absolute feedback linearization control based on the universal approximation theorem [18] can be expressed as

(26) $$\begin{array}{c} P_{\text{con}}^{*}=P_{fz}^{*}\left(\alpha^{*},\xi \right)+\epsilon \\ =\alpha^{*T}\xi +\epsilon , \end{array}$$

where *ϵ* depicts the approximation error described as

(27) $$\begin{array}{c} \epsilon =P_{\text{con}}^{*}-P_{fz}^{*}\left(\alpha^{*},\xi \right), \end{array}$$

To realize the perfect feedback linearization control *P*_con_^*∗*^, the fuzzy control law *P*_*fz*_^*∗*^(*α*^*∗*^, *ξ*) can be approximated as follows:

(28) $$\begin{array}{c} {\hat{P}}_{fz}\left(\hat{\alpha },\xi \right)={\hat{\alpha }}^{T}\xi , \end{array}$$

where $\hat{\alpha }$ is the estimation of *α*^*∗*^. Despite the capacity that *P*_*fz*_ will strive to approach *P*_con_^*∗*^, there is always some residual error between *P*_*fz*_ and *P*_con_^*∗*^. This error will be minimized by augmenting the sliding mode-based discontinuous switching term *P*_*sw*_ in the control expression described as

(29) $$\begin{array}{c} P_{\text{con}}={\hat{P}}_{fz}\left(\hat{\alpha },\xi \right)+P_{\text{sw}}, \end{array}$$

where

(30) $$\begin{array}{c} P_{sw}=-K\text{sign}\left(s\left(t\right)\right), \end{array}$$

The switching control law is intended to minimize the error between the designed fuzzy law ${\hat{P}}_{fz}$ and perfect feedback linearization control law *P*_con_^*∗*^. The resultant control law *P*_con_ given by (29) leads to the robust control approach to achieve smooth and precise tracking performance even if the system under consideration subjects to high degree of uncertainty.

The article "Adaptive Fuzzy Sliding Mode Control of a Pressure-Controlled Artificial Ventilator" was published in 2021. Journal: J Healthc Eng.

**Theorem 1 .**

Consider the mechanical ventilator system given by (38), the control law given by (29), with fuzzy control element ${\hat{P}}_{fz}$ given by (28) and the switching control element *P*_*sw*_ given by (30), ensures the finite-time stability while tracking error converges to zero.

**Proof**

To prove the finite-time stability, the expressions of perfect feedback linearization control law given by (20) and sliding mode dynamics given by (22) are solved for *P*_con_^*∗*^, which yields the following expression:

(31) $$\begin{array}{c} P_{\text{con}}^{*}=\frac{1}{g\left(x,t\right)}\left[g\left(x,t\right)P_{\text{con}}-\dot{s}\left(t\right)\right]. \end{array}$$

Substituting the control law *P*_con_ given by (29) in (31) yields the following sliding mode dynamics:

(32) $$\begin{array}{c} \dot{s}\left(t\right)=g\left(x,t\right)\left[{\hat{P}}_{fz}+P_{sw}-P_{\text{con}}^{*}\right]. \end{array}$$

Choose the following Lyapunov candidate function:

(33) $$\begin{array}{c} V_{1}\left(s\left(t\right),\tilde{\alpha }\right)=\frac{1}{2}s^{2}\left(t\right)+\frac{1}{2\gamma_{1}}{\tilde{\alpha }}^{T}\tilde{\alpha }, \end{array}$$

where *γ*_1_ is a positive constant. Taking the time derivative of *V*_1_ yields the following equation:

(34) $$\begin{array}{c} \begin{array}{cc} {\dot{V}}_{1}\left(s\left(t\right),\tilde{\alpha }\right) & =s\left(t\right)\dot{s}\left(t\right)+\frac{g}{\gamma_{1}}{\tilde{\alpha }}^{T}\dot{\tilde{\alpha }}, \end{array} \end{array}$$

(35) $$\begin{array}{c} =s\left(t\right)g\left({\hat{P}}_{fz}+P_{sw}-P_{\text{con}}^{*}\right)+\frac{g}{\gamma_{1}}{\tilde{\alpha }}^{T}\dot{\tilde{\alpha }}, \end{array}$$

(36) $$\begin{array}{c} =s\left(t\right)g\left({\tilde{\alpha }}^{T}\xi +P_{sw}-\epsilon \right)+\frac{g}{\gamma_{1}}{\tilde{\alpha }}^{T}\dot{\tilde{\alpha }}, \end{array}$$

(37) $$\begin{array}{c} =g{\tilde{\alpha }}^{T}\left\{s\left(t\right)\xi +\frac{1}{\gamma_{1}}\dot{\tilde{\alpha }}\right\}+s\left(t\right)g\left(P_{sw}-\epsilon \right). \end{array}$$

To ensure the finite-time stability of the closed-loop system, let us define the adaptive law as follows:

(38) $$\begin{array}{c} \dot{\tilde{\alpha }}=\dot{\hat{\alpha }}=-\gamma_{1}s\left(t\right)\xi . \end{array}$$

Placing the expression of *P*_*sw*_ given by (30) leads to the following expression of ${\dot{V}}_{1}$:

(39) $$\begin{array}{c} {\dot{V}}_{1}\left(s\left(t\right),\tilde{\alpha }\right)=-K\left|s\left(t\right)\right|g-\epsilon s\left(t\right)g\leq -K\left|s\left(t\right)\left|g-\right|\epsilon s\left(t\right)\right|g \end{array}$$

(40) $$\begin{array}{c} =-\left(K+\left|\epsilon \right|\right)\left|s\left(t\right)\right|g\leq 0. \end{array}$$

Considering that the sliding surface *s* is uniformly continuous, the Lyapunov stability is guaranteed by negative semidefiniteness of ${\dot{V}}_{1}\left(s\left(t\right),\tilde{\alpha }\right)$. Asymptotic stability of the closed-loop system follows from Barbalat's lemma [43], such that $\left(s\left(t\right),\tilde{\alpha }\right)⟶\left(0,0\right)$ as *t*⟶*∞*.

The article "Adaptive Fuzzy Sliding Mode Control of a Pressure-Controlled Artificial Ventilator" was published in 2021. Journal: J Healthc Eng.

**Proof**

The next objective is to find the appropriate value of sliding mode gain *K*, which needs to be smooth enough in order to avoid undesirable chattering phenomenon. If *K* is made small, it will reduce chattering, but it may lead to inferior tracking performance. Hence, it would be preferable to make the sliding mode gain adaptively to achieve better tracking accuracy and closed-loop stability. By replacing *K* by $\hat{K}$, the equation of the switching (discontinuous) control law is described as

(41) $$\begin{array}{c} {\hat{P}}_{sw}=-\hat{K}\left(t\right)\text{sign }\left(s\left(t\right)\right), \end{array}$$

where $\hat{K}$ is the estimation of *K*. Based on this, the control law given by (29) is written as

(42) $$\begin{array}{c} P_{\text{con}}={\hat{P}}_{fz}\left(\hat{\alpha },\xi \right)-\hat{K}\left(t\right)\text{sign }\left(s\left(t\right)\right). \end{array}$$

**Theorem 2 .**

Consider the mechanical ventilator system given by (38), the control law given by (42), comprising fuzzy-based controller ${\hat{P}}_{fz}$ and switching control element *P*_*sw*_, guarantees that the closed-loop system is asymptotically stable in the sense of Lyapunov and the system follows the desired reference output in presence of modeling uncertainties and disturbances.

**Proof**

Define the estimation error of sliding mode gain as

(43) $$\begin{array}{c} \tilde{K}\left(t\right)=\hat{K}\left(t\right)-K. \end{array}$$

Now, consider the Lyapunov energy function *V*_2_ as

(44) $$\begin{array}{c} V_{2}\left(s\left(t\right),\tilde{\alpha },\tilde{K}\right)=\frac{1}{2}s^{2}\left(t\right)+\frac{1}{2\gamma_{1}}g{\tilde{\alpha }}^{T}\tilde{\alpha }+\frac{1}{2\gamma_{2}}{\tilde{K}}^{2}, \end{array}$$

where *γ*_2_ is the positive gain constant. The time derivative of *V*_*s*_ along the error trajectory given by (44) is

(45) $$\begin{array}{c} {\dot{V}}_{2}\left(s\left(t\right),\tilde{\alpha },\tilde{K}\right)=s\left(t\right)\dot{s}\left(t\right)+\frac{g}{\gamma_{1}}{\tilde{\alpha }}^{T}\dot{\tilde{\alpha }}++\frac{g}{\gamma_{2}}\tilde{K}\dot{\tilde{K}}\\ =g\left(\right){\tilde{\alpha }}^{T}\left(s\left(t\right)\xi +\frac{1}{\gamma_{1}}{\dot{\hat{\alpha }}}^{T}\right)+s\left(t\right)g\left(P_{sw}-\epsilon \right)+\frac{g}{\gamma_{2}}\tilde{K}\dot{\tilde{K}}\\ =-\hat{K}\left(t\right)|s\left(t\right)|g-\epsilon s\left(t\right)g+\frac{g}{\gamma_{2}}\left(\hat{K}\left(t\right)-K\right)\dot{\hat{K}}\left(t\right). \end{array}$$

To establish asymptotic convergence of the tracking error such that ${\dot{V}}_{2}\leq 0$, the estimation law is defined as

(46) $$\begin{array}{c} \dot{\hat{K}}\left(t\right)=\gamma_{2}\left|s\left(t\right)\right|, \end{array}$$

By substituting the expression of $\dot{\hat{K}}$, the time derivative of *V*_2_ given by (45) can be written as

(47) $$\begin{array}{c} \begin{array}{cc} {\dot{V}}_{2}\left(s\left(t\right),\tilde{\alpha },\tilde{K}\right) & =-\hat{K}\left(t\right)\left|s\left(t\right)\right|g-\epsilon s\left(t\right)g+\left(\hat{K}\left(t\right)-K\right)\left|s\left(t\right)\right|g \end{array}, \end{array}$$

(48) $$\begin{array}{c} =\epsilon s\left(t\right)g-K\left|s\left(t\right)\right|g\leq \left|\epsilon s\left(t\right)\right|g-K\left|s\left(t\right)\right|g, \end{array}$$

(49) $$\begin{array}{c} =\left(K-\left|\epsilon \right|\right)\left|s\left(t\right)\right|g\leq 0. \end{array}$$

Negative semidefiniteness of ${\dot{V}}_{2}\left(s\left(t\right),\tilde{\alpha },\tilde{K}\right)$ implies the Lyapunov stability of the system equilibrium $\left(s\left(t\right),\tilde{\alpha },\tilde{K}\right)=\left(0,0,0\right)$. Asymptotic stability follows from Barbalat's lemma, see, e.g., [43].

The article "Adaptive Fuzzy Sliding Mode Control of a Pressure-Controlled Artificial Ventilator" was published in 2021. Journal: J Healthc Eng.

The AFSMC structure given by (42) encompassing fuzzy and switching control elements to track the targeted pressure commands is illustrated in Figure 3.

## 4. Numerical Simulations

The practical applicability of AFSMC for pressure control in the simulated mechanical ventilation system is demonstrated in this section. The nominal values of the system parameters of artificial mechanical ventilator are chosen as *R*_Lung_=0.005mbar/mL/s, *R*_Leak_=0.06mbar/mL/s, and *R*_hose_=0.0045mbar/mL/s. For computer simulation, the targeted airway pressure is set to be 0.30 mbar. Three control methodologies—AFSMC, SMC, and PID—are implemented in order to illustrate the performance comparison. The tradeoff between faster convergence toward the desired values, settling time, and overshoot in the response curves of three control strategies is shown in Figure 4.

The superiority of AFSMC over conventional PID and SMC is clearly observed through simulation results. The AFSMC demonstrates smooth tracking performance with small tracking error compared with its counterparts. Furthermore, the key performance indices of AFSMC, SMC, and PIC control schemes in response to the square wave input of targeted airway pressure are listed in Table 1. It is apparent that no overshoot has been observed in all the simulation cases.

To quantify the tracking performance, the time histories of the magnitude of residual error of the control methodologies under consideration are illustrated in Figure 5, which reveals that the AFSMC scheme adequately follows the desired pressure curve.

## 5. Robust Analysis

In this section, to gain a qualitative insight of the robustness characteristic and sensitivity of AGDI control, a realistic scenario is exercised by introducing 20% random variations in the parameters of artificial ventilator system such as *R*_*l*_, *R*_*h*_, and *R*_leak_. The magnitude of ventilator parameter lung compliance *C*_lung_, which determines the change in lung volume per change in trans-pulmonary pressure, is also varied as its value is not constant and changes accordingly with respect to the lung's volume. Computer simulation is performed by commanding the targeted airway pressure of 0.30 mbar for the artificial ventilator. The response curves of targeted and achieved airway pressure are depicted in Figure 6, which reveals effective tracking of pressure commands along with faster convergence toward the reference value. The corresponding control input command is shown in Figure 7, which is very much realizable. From simulation results, it is concluded that the AGDI control is made adaptive and robust against parametric variations and proven to be effective and feasible for its applications to real-world systems.

## 6. Conclusion

The paper presents the design of AFSMC for smooth tracking of targeted pressure curves of the mechanical ventilation systems. For performance evaluation, along with AFSMC, two other control approaches (PID and SMC) are also implemented and their performances have been verified in terms of convergence toward the targeted pressure curves of the artificially ventilated human respiratory system. The AFSMC approach reveals better pressure tracking performance by adjusting the ventilator output pressure curves adaptively in comparison with SMC and PID. In future work, the presented approach can further be checked and verified through numerical simulation as well as experimental investigations for a more complex human lung artificially ventilated system.

The article "Adaptive Fuzzy Sliding Mode Control of a Pressure-Controlled Artificial Ventilator" was published in 2021. Journal: J Healthc Eng.

## Figures and Tables

**Figure 1:** Blower-hose-patient system.

**Figure 2:** Singleton control.

**Figure 3:** AFSMC block diagram.

**Figure 4:** Airway pressure.

**Figure 5:** Residual error.

**Figure 6:** Airway pressure.

**Figure 7:** Control input.

**Table 1:** Performance comparison.

Parameters	AFSMC	SMC	PID
Rise time, *sec*	2.129	2.729	3.530
Settling time, *sec*	3.640	4.357	5.522

## Data Availability

No data were used to support this study.
